# Brain Diffusion Weighted Imaging Study of Mongolian Idiopathic Epilepsy

**DOI:** 10.1155/2022/6978116

**Published:** 2022-11-28

**Authors:** Pengfei Zhao, Xueying Ma, Chao Ban, Yang Gao, Pengfei Qiao

**Affiliations:** Department of Radiology, Affiliated Hospital of Inner Mongolia Medical University, Huhhot 010050, China

## Abstract

**Objective:**

To evaluate the effectiveness of diffusion-weighted imaging in the assessment of idiopathic epilepsy in Mongolian.

**Methods:**

One hundred Mongolian idiopathic epilepsy patients were enrolled as the observation group and 100 healthy Mongolian volunteers as the control group. All the subjects underwent routine MRI, diffusion kurtosis imaging (DKI), and intra-voxel incoherent motion (IVIM) examination on a 3.0 T scanner. Mean kurtosis (MK), mean diffusivity (MD), fractional anisotropy (FA), true water molecular diffusion coefficient (*D*), mean diffusion coefficient (MD), pseudo-diffusion coefficient (*D∗*), and perfusion fraction (*f*) of each region of interest in the brain were measured. Count data were expressed as rates, and the chi-square test was performed for comparison between groups. Measurement data were first assessed by a normality test, and the *t* test for independent samples was performed for comparison between groups if they met the normal distribution; for non-normal distribution, the Mann-Whitney *U* test was performed for comparison between groups. A ROC curve analysis was performed to test the effectiveness of each parameter.

**Results:**

MK values of the hippocampus, thalamus, and white matter of the temporal lobe in the observation group were significantly higher than those in the control group, while *D* and F values were significantly lower (all *P* < 0.05). ROC curve analysis showed that MK, *D*, and F values of the hippocampus, thalamus, and white matter of the temporal lobe had moderate to good diagnostic efficacy for idiopathic epilepsy (AUC = 0.617–0.749, all *P* < 0.001).

**Conclusion:**

DKI and IVIM can more accurately represent the abnormal changes of brain tissue in patients with epilepsy, and it may have important implications for the clinical diagnosis of Mongolian epileptic patients.

## 1. Introduction

Idiopathic epilepsy is a chronic neurological disorder characterized by sudden, transient, and recurrent central nervous system dysfunction caused by super-synchronous abnormal neuronal discharges in the brain, the pathogenesis of which has not been fully elucidated and may be related to genetic factors. The disease mainly occurs in children and young adults with complex pathophysiological mechanisms and diverse clinical manifestations, and so far, drugs are the most common and primary treatment [1].

The results of a bioinformatics study by some scholars, screening identified 25-key differentially expressed genes (DEGs), including TREML3P, KCNJ15, ORM1, CCL3, and RNA28S5. These DEGs were involved in biological processes such as immune response, inflammatory response, and chemotaxis. Meanwhile, the molecular functions were focused on peroxidase activity, chemokine activity, etc., while KEGG pathway enrichment analysis showed that DEGs were mainly involved in cytokine-cytokine receptor interaction, Toll-like receptor signaling pathway, and chemokine signaling pathway [2]. These important key DEGs may be involved in the development of idiopathic epilepsy through multiple signaling pathways and complex mechanisms. The epidemiological studies on idiopathic epilepsy in Inner Mongolia are few, mostly focusing on urban-rural differences in the onset of idiopathic epilepsy and later interventions, and most of the studies did not focus on ethnic differences. Therefore, the present study focuses on the imaging diagnosis of idiopathic epilepsy in Mongolian ethnic groups, which is innovative in China.

The main methods applied in clinical diagnosis and therapeutic evaluation of epilepsy are electroencephalogram (EEG) [3, 4], positron emission computed tomography (PET-CT), single photon emission computed tomography (SPECT), and magnetic resonance imaging (MRI) [5]. EEG has a high sensitivity in seizures, but its diagnostic value is greatly reduced in non-epileptic seizures. PET-CT and SPECT are too expensive to be not popularized [6, 7]. Conventional MRI is difficult to display the microscopic structure of the brain, and it is difficult to find the epileptogenic foci in the cerebellum, and it cannot well locate the epileptogenic foci. While MRI has made great methodological progress in recent years, the successive emergence of intro-voxel incoherent movement (IVIM) and diffusion kurtosis imaging (DKI) techniques have achieved a leap from macroscopic imaging to microscopic imaging and even functional evaluation [8–10]. DKI is an emerging diffusion imaging technique that extends the traditional diffusion tensor imaging (DTI) to capture the non-Gaussian diffusion properties of water molecules in biological tissues. DKI represents the complexity of tissue microstructure and the corresponding pathophysiological changes in diseases. In the present study, the MK value, FA value, and MD values were selected to analyze whether there were subtle structural changes in the brain tissue of Mongolian idiopathic epilepsy. MK is an important parameter of DKI, which is the average of multiple *b* values with the same gradient direction, and its magnitude reflects the complexity of tissue structure. The MD value is the mean value of the diffusion amplitude in each direction, demonstrating the size or degree of diffusion of water molecules in a voxel. The FA value describes the degree of anisotropic diffusion of water molecules, and the closer the FA value is to 1, the more the diffusion direction of water molecules tends to the direction of nerve fiber alignment [11–13]. The parameters obtained from the IVIM biexponential model are perfusion parameters *D∗* and *f* and diffusion parameter *D*. The value of *D∗* captures the microcirculatory perfusion-related components of the capillary network; the value of *f* explains the percentage of diffusion-related components of the microcirculatory perfusion in the total diffusion; and the value of *D* mirrors the water molecules in the real tissue. There are many studies on IVIM imaging in glioma grading at home and abroad, and IVIM could be used as a non-invasive predictor of preoperative grading of glioma [14–16]. Based on these new techniques, we attempted to assess the occurrence and development of epilepsy using brain diffusion imaging. Considering that genetics plays an important role in the pathogenesis of idiopathic epilepsy, this study selected a Mongolian population for the study, with the main purpose of observing the brain diffusion imaging features of idiopathic epilepsy and providing clinical value for the diagnosis of idiopathic epilepsy based on observed data.

## 2. Material and Methods

### 2.1. Study Object

This prospective study is based on 100 patients with first-episode idiopathic epilepsy and 100 healthy volunteers. The observation group of 100 patients with first-onset idiopathic epilepsy, who were all Mongolian direct blood relatives of three generations admitted to our hospital from December 2017 to December 2019. All cases were classified as seizures and syndromes according to the International League Against Epilepsy (ILAE) 2017 diagnostic criteria and judged as idiopathic epilepsy, and the enrolled cases were strictly controlled as “first episode [17]. In all cases, a physician with clinical experience and above took a medical history and combined it with the corresponding EEG changes to exclude (1) perinatal brain injury; (2) other lesions of the central nervous system; (3) neonatal convulsions and febrile convulsions; (4) family history of epilepsy, febrile convulsions, migraine, and other neurological disorders, and finally confirmed the clinical stage. The study subjects had no abnormalities on a neurological specialist examination and were free of serious somatic diseases and complications. There were no significant structural abnormalities on the routine brain MRI. One hundred healthy volunteers matched for ethnicity, age, sex, and years of education were recruited as a control group among the population admitted for physical examination at the same time. The study was approved by the Ethics Committee of the Affiliated Hospital of Inner Mongolia Medical University (S.2019014), and all study subjects voluntarily signed the informed consent form.

### 2.2. Clinical Brain Diffusion Imaging Examination Methods

After the patients' first seizure (through careful history taking, it was confirmed that the patient did not have any previous epileptic symptoms and no significant organic lesions were seen on imaging), brain diffusion-weighted imaging (DWI) was performed using a Discovery MR 750 3.0 T superconducting type magnetic resonance instrument provided by GE Healthcare (Chicago, IL, USA). An 8 neuro vascular (NV)-Head coil was used with the subject's eyes tightly closed and the head held stationary, and the examination sequence included axial T1WI, TR 3207 ms, TE 25.2 ms, ETL 8; axial T2WI, TR 8753 ms, TE 95.6 ms, ETL 31; and axial FLAIR, TR 9000 ms, TE 91.5 ms, ETL 18. IVIM, *b* values (10, 25, 50, 75, 100, 150, 200, 400, 800, 1000, 1200, 1500 s/mm^2^), TR 3500 ms, TE Minimum, FOV 260 mm × 260 mm, layer thickness 5 mm, layer spacing 1 mm, number of scanned layers 22; diffusion kurtosis imaging (DKI), b-values (0, 1000, 2000 s/mm^2^), diffusion-sensitive gradient field applied in 50 directions, b-value 0 scanned 2 times, TR 3200 ms, TE Minimum, FOV 240 mm × 240 mm, layer thickness 5 mm, layer spacing 0 mm, and the number of layers scanned 30 times. The scanned DKI and IVIM sequence raw DICOM data were transferred to the workstation, and the images were processed using the processing software of the functool package provided by GE Healthcare (Chicago, IL, USA). Twelve brain regions were selected as regions of interest (ROIs), namely, bilateral hippocampal head, caudate head, thalamus, white matter of frontal, temporal, and parietal lobes [18, 19]. Under the guidance of experts, two doctors with 5 years of working experience delineated each brain area 3 times, the size of the circular ROI was 2.0–3.0 mm^2^ (Table 1). The mean kurtosis (MK) values, mean diffusion rate (MD) values, fractional anisotropy (FA) values, true water molecule diffusion coefficients (*D*), pseudo-diffusion coefficient (*D*^*∗*^), and perfusion fraction (*f*) were measured for each ROI. Then the mean values of each parameter were calculated for each brain region. *D*, *D*^*∗*^, and *f* plots were derived by using a biexponential intra-voxel incoherent motion (IVIM) analysis [20]:

(1) $$\begin{array}{c} \frac{S\left(b\right)}{S\left(0\right)}=\left[f\cdot \;\exp\;\left(-b\cdot D^{*}\right)\right]+\left[\left(1-f\right)\cdot \;\exp\;\left(-b\cdot D\right)\right]\text{.} \end{array}$$

MD, FA, and MK plots were calculated based on the DKI dataset [20]:

(2) $$\begin{array}{c} \frac{S\left(b\right)}{S\left(0\right)}=\exp\;\left(-b\cdot D_{app}＋\frac{1}{6}b^{2}\cdot D_{app}^{2}\cdot K_{app}\right)\text{,}\\ FA=\sqrt{\frac{{\left(\lambda_{1}-\lambda_{2}\right)}^{2}＋{\left(\lambda_{2}-\lambda_{3}\right)}^{2}+{\left(\lambda_{1}-\lambda_{3}\right)}^{2}}{2\left(\lambda_{1}^{\;2}＋\lambda_{2}^{2}＋\lambda_{3}^{2}\right)}}\text{.} \end{array}$$

### 2.3. Statistical Analysis

The statistical software SPSS 22.0 was conducted to analyze the data; the count data were expressed as rates, and the chi-square test was performed for comparison between groups; the measurement data were first assessed by the normality test. FA, MD, and MK values were normally distributed and expressed as mean ± standard deviation; an independent sample *t*-test was performed for comparison between two groups. *D∗*, *D*, and *f* values were not normal distribution and were expressed as Median ± Quartiles, and Mann-Whitney *U* test was performed for comparison between groups; ROC curve was used for predictive analysis of FA, MD, MK, *D∗*, *D*, and *f* values. *P* < 0.05 was considered significantly statistical difference.

## 3. Result

### 3.1. Participants Characteristics

Clinical and demographic data for subjects such as gender, age, body mass index (BMI), handedness, and education were matched (*P* > 0.05) (Table 2).

### 3.2. Comparison of Brain Diffusion Weighted Imaging Parameters between Patients with Idiopathic Epilepsy and Healthy Volunteers in Mongolian

Between the patients and the healthy volunteers, there were significant differences observed in 3 parameters in 3 brain regions, named MK, *D,* and *f* in the hippocampus, thalamus, and white matter of the temporal lobe, respectively. Compared to the lower *D* and *f* values, the MK values were greater in the three brain regions of the patient group, with statistically significant differences compared to the control group (MK: hippocampus: *t* = 3.183, *P*=0.001; thalamus: *t* = 3.065, *P*=0.001; temporal lobe: *t* = 2.988, *P*=0.002. D : Hippocampus: *Z* = 32.889, *P*=0.015; thalamus: *Z* = 29.578, *P*=0.019; temporal lobe: *Z* = 32.001, *P*=0.016. *f*: Hippocampus: *Z* = 29.011, *P*=0.020; thalamus: *Z* = 28.885, *P*=0.025; temporal lobe: *Z* = 28.998, *P*=0.022). Details are shown in Table 3 and Figures 1 and 2.

### 3.3. Clinical Application Value of Brain Diffusion Weighted Imaging Parameters for the Diagnosis of Mongolian Idiopathic Epilepsy

ROC curves were conducted to analyze the clinical diagnostic value of MK, *D*, and *f* values for idiopathic epilepsy, and the results showed that MK, *D*, and *f* values of the hippocampal region, thalamus, and temporal lobe white matter had moderate to good diagnostic efficacy for idiopathic epilepsy (AUC = 0.617–0.749, all *P* < 0.001), and the sensitivity of their optimal working point was 49.0%–72.0%, and the specificity was 56.0% to 91.0%, as shown in Figure 3 and Table 4.

## 4. Discussion

The clinical diagnosis of epilepsy mainly relies on clinical manifestations, neurophysiology, and imaging examinations, and the lack of obvious organic changes in primary epilepsy is a major limitation in pathological studies [21]. In our previous study, it has been confirmed that the multimodal MRI features of the Wistar rat epilepsy model are highly consistent with the histopathological features of the brain and confirmed that the changes in multimodal MRI parameters FA, MD, and MK values laterally demonstrate the changes in pathological parameters [22]. In this study, we further improved the multimodal MRI diagnostic system by incorporating IVIM technology into the system as well and analyzed the application value of the system from both clinical and animal models.

In the present study, diffusion-weighted imaging was applied to evaluate Mongolian idiopathic epilepsy, and considering the importance of genetics in the pathogenesis of primary epilepsy, patients with first episode primary epilepsy who were three generations of direct relatives of Mongolian descent were selected as the primary study population, while matching healthy volunteers for ethnicity, gender, and age. Significant differences were found between the case group and the healthy volunteers in three parameters in three brain regions: MK, *D*, and *f* values in the hippocampal region, thalamus, and temporal lobe white matter; MK values were higher and *D* and *f* values were lower in three brain regions in the patient group, and the differences were statistically significant compared with the control group. The MK, *D*, and *f* values of the hippocampus, thalamus, and temporal lobe white matter were found to have good diagnostic efficacy for primary epilepsy. Previous studies have suggested that the thalamus and hippocampus are closely related to higher cognitive brain functions such as learning and memory, and patients with idiopathic epilepsy have varying degrees of sclerosis in the hippocampal region, as evidenced by volume reduction, widening of cell gaps, and neuronal loss [23–26]. The diagnostic results of 147 cases of temporal lobe epilepsy by Zhang Xiaona showed that the detection rate of hippocampal sclerosis was as high as 92.52%, including bilateral sclerosis at 44.85% and unilateral sclerosis at 57.35%. It is evident that the hippocampus plays an important role in the pathogenesis of epilepsy [27]. Another study pointed out that hippocampal sclerosis was often accompanied by localized temporal lobe white matter abnormalities [28], and the results of the present study supported this view.

The MK value is the main parameter of the DKI technique, which is the only technique currently available for non-invasive detection of tissue microstructural information in vivo [29]. It is indicated that the MK value is the average of the dispersion kurtosis of water molecules along each spatial direction, which is mainly used to respond to the complexity of local structures, and its size reveals the complexity of the tissue structure, with larger values indicating more restricted dispersion, very sensitive to microstructural changes in the white matter of the brain, independent of the spatial orientation of the tissue structure, and high stability. In contrast, the most common pathological changes in epilepsy are neuronal loss and reactive glial cell proliferation with altered extracellular gaps leading to changes in water molecule movement [30, 31]. Therefore, DKI imaging is usually used to show epileptic foci [32]. In our study, MK values were found to be higher in epileptic patients than those in healthy volunteers, due to the pathological changes in primary epilepsy characterized by local sclerosis, neuronal loss, reduced tissue homogeneity, and increased microstructural complexity.

*D* value and *f* value are the main parameters of the IVIM technique, where the *D* value mainly responds to the true diffusion of water molecules and *f* value mainly responds to the percentage of microcirculatory perfusion components [11]. In this study, both *D* and *f* values were found to be lower in epileptic patients than those in healthy volunteers, which is inextricably linked to their pathological alterations. Recurrent seizures can lead to ischemic hypoxic damage to the brain tissue and the production of large amounts of reactive oxygen radicals, which leads to a local perfusion deficit and lower *f* values [23].

The results of the final ROC curve analysis confirmed the good diagnostic efficacy of MK, *D*, and *f* values for primary epilepsy (AUC = 0.617–0.749); it suggested that MK, *D*, and *f* values have sufficient clinical diagnostic value to aid in the adjunctive diagnosis of idiopathic epilepsy. Perhaps the pathophysiological changes reflected by MK, *D*, and *f* are consistent with the pathophysiological changes of epilepsy, as described above. Therefore, the area under the ROC curve is the largest.

However, there are some limitations in this paper; for example, there are too many *b* values in IVIM, which increases the scanning time and motion artifacts. We will optimize the sequence and reduce the *b* value in later research, so as to shorten the scanning time without affecting the research results. Although similar research was carried out earlier in this study, 8 neurovascular (NV) head coils were also used, and better DKI and IVIM images were archived. Based on some relevant literature in China, the present study used an 8NV head coil to collect DKI and IVIM data. But 24 or 32 will be selected to obtain higher quality data in further research. In an era of the vigorous development of artificial intelligence (AI), we will try to introduce AI for correlation analysis in the future.

## 5. Conclusion

In conclusion, this study applied certain parameters of DWI MRI to describe microscopic changes in idiopathic epilepsy, and it provided a reliable diagnostic basis during the non-ictal phase of idiopathic epilepsy.

## Figures and Tables

**Figure 1:** MRI images of three brain regions in Mongolian idiopathic epilepsy patients (GE advantage workstation 4.6); (a) pseudo-color map of MK values of three brain regions in the observation group; (b) pseudo-color map of *D* values of three brain regions in the observation group; (c) pseudo-color map of *f* values of three brain regions in the observation group. 1: hippocampus; 2: thalamus; 3: temporal lobe.

**Figure 2:** MRI images of three brain regions in Mongolian control group (GE advantage workstation 4.6); (d) pseudo-color map of MK values of three brain regions in the control group; (e) pseudo-color map of *D* values of three brain regions in the control group; (f) pseudo-color map of *f* values of three brain regions in the control group. 1: hippocampus; 2: thalamus; 3: temporal lobe.

**Figure 3:** ROC curve of MK value, *D* value, and *f* value to diagnose the onset of Mongolian idiopathic epilepsy.

**Table 1:** Interobserver variability in measurements of 100 randomly selected patients.

Parameter	ICC	*P* value
MK	0.705	0.009
MD	0.713	0.009
FA	0.579	0.011
*D*	0.628	0.010
*D∗*	0.518	0.013
*f*	0.580	0.011

*Note.* ICC: intraclass correlation coefficient, MK: mean kurtosis, MD: mean diffusion, FA: fractional anisotropy, *D*: true water molecule diffusion coefficients, *D∗*: pseudo-diffusion coefficient (*D∗*), *f*: perfusion fraction.

**Table 2:** Demographic and clinical characteristics of patients with idiopathic epilepsy (*n* = 100) and healthy volunteers in Mongolian (HVs) (*n* = 100).

Items		Observation group (*n* = 100)	Control group (*n* = 100)	Statistical values	*P* values
Gender	Male	53	54	0.02	0.89
	Female	47	46		

Handedness	Right	100	100	0	1
	Left	0	0		

Age (years)		26.6 ± 4.3	26.0 ± 3.9	2.11	0.86
BMI (kg/m^2^)		22.95 ± 3.68	23.24 ± 2.43	1.68	0.56
Education (years)		13.7 ± 2.6	14.0 ± 1.9	0.24	0.79

**Table 3:** Comparison of brain diffusion weighted imaging parameters between two groups.

Groups	Brain regions	FA values	MD values	MK values	*D* values (× 10^−3^ mm/s)	*D∗* values (× 10^−3^ mm/s)	*f* values (%)
Observation group	Hippocampus	0.14 ± 0.03	0.91 ± 0.10^*∗*^	0.46 ± 0.07^*∗*^	0.791 ± 0.410^*∗*^	3.662 ± 2.450	26.2 ± 17.1^*∗*^
	Caudate head	0.27 ± 0.07	0.85 ± 0.07	0.43 ± 0.04	0.851 ± 1.066	3.852 ± 2.346	24.1 ± 19.0
	Thalamus	0.30 ± 0.05	0.88 ± 0.06	0.67 ± 0.08^*∗*^	0.668 ± 0.377^*∗*^	3.745 ± 2.804	25.1 ± 20.1^*∗*^
	Frontal white matter	0.43 ± 0.08	0.94 ± 0.07	0.75 ± 0.09	0.636 ± 0.483	4.005 ± 2.866	27.0 ± 19.4
	Temporal lobe white matter	0.15 ± 0.03	0.88 ± 0.10	0.57 ± 0.08^*∗*^	0.620 ± 0.454^*∗*^	3.662 ± 2.450	27.3 ± 22.0^*∗*^
	Parietal white matter	0.33 ± 0.09	1.00 ± 0.10	0.85 ± 0.10	0.609 ± 0.511	3.641 ± 1.500	28.5 ± 20.0
Control group	Hippocampus	0.15 ± 0.04	0.95 ± 0.12	0.41 ± 0.06	0.952 ± 0.357	4.065 ± 0.950	31.2 ± 21.3
	Caudate head	0.29 ± 0.06	0.84 ± 0.09	0.42 ± 0.08	0.950 ± 0.471	3.852 ± 3.346	25.5 ± 18.4
	Thalamus	0.30 ± 0.06	0.86 ± 0.05	0.71 ± 0.09	0.705 ± 0.952	3.778 ± 2.522	28.8 ± 20.9
	Frontal white matter	0.44 ± 0.09	0.95 ± 0.08	0.81 ± 0.10	0.625 ± 0.308	4.112 ± 1.187	28.2 ± 20.7
	Temporal lobe white matter	0.16 ± 0.04	0.92 ± 0.11	0.53 ± 0.08	0.705 ± 0.391	4.085 ± 4.450	31.5 ± 30.4
	Parietal white matter	0.35 ± 0.10	1.02 ± 0.11	0.83 ± 0.11	0.766 ± 0.610	3.854 ± 0.741	30.5 ± 19.0

*Note.* ^*∗*^ represents *P* < 0.05.

**Table 4:** Results of ROC curve of MK value, *D* value, and *f* value to diagnose the onset of Mongolian idiopathic epilepsy.

Items	AUC	*P*	95% CI	Best working point	Sensitivity (%)	Specificity (%)
MK values						
Hippocampus	0.617	<0.001	0.546–0.685	0.485	66.0	57.0
Thalamus	0.625	0.001	0.558–0.696	0.806	67.0	56.0
Temporal lobe white matter	0.728	0.001	0.661–0.788	32.1%	55.0	84.0
*D* values						
Hippocampus	0.723	≤0.001	0.656–0.784	0.677	66.0	73.0
Thalamus	0.672	≤0.001	0.603–0.737	0.700	65.0	66.0
Temporal lobe white matter	0.682	≤0.001	0.613–0.746	29.5%	49.0	76.0
*F* Values						
Hippocampus	0.657	≤0.001	0.586–0.722	0.595	49.0	76.0
Thalamus	0.615	0.004	0.543–0.682	0.806	35.0	91.0
Temporal lobe white matter	0.749	≤0.001	0.683–0.808	28.4%	72.0	65.0

## Data Availability

The authors confirm that the data supporting the findings of this study are available within the article.
